The article "Kinematic analysis and process optimization of root-cutting systems in field harvesting of garlic based on computer simulation technology" was published in 2023. Journal: Front Plant Sci.

# Kinematic analysis and process optimization of root-cutting systems in field harvesting of garlic based on computer simulation technology

**DOI:** 10.3389/fpls.2023.1168900

**Published:** 2023-08-22

**Authors:** Zhaoyang Yu, Mingjin Yang, Zhichao Hu, Fengwei Gu, Baoliang Peng, Yanhua Zhang, Ke Yang

**Affiliations:** ^1^ College of Engineering and Technology, Southwest University, Chongqing, China; ^2^ Nanjing Institute of Agricultural Mechanization, Ministry of Agriculture and Rural Affairs, Nanjing, China; ^3^ Key Laboratory of Modern Agricultural Equipment, Ministry of Agriculture and Rural Affairs, Nanjing, China

**Keywords:** garlic field harvesting, floating root-cutting, computer simulation, virtual orthogonal test, fuzzy comprehensive evaluation, root excision rate

## Abstract

**Introduction:**

Root cutting is an important process in garlic field harvesting but is the weakest link in the full mechanization of garlic production. To improve the current situation of technological backwardness and poor operational quality of mechanized garlic root-cutting in the main garlic-producing regions of China, this study combined the physical characteristics and agronomic requirements of garlic plants, and proposed an innovative floating root-cutting technology for garlic combine harvesters that enables the top alignment of bulb, adaptive profiling floating of cutter, and embedded cutting of roots.

**Methods:**

Through the kinematic analysis of the floating cutting process, the coordinate equations of the initial contact point of the bulb, the mathematical model of the floating displacement of the cutting component. Using computer simulation techniques, the dynamic simulation study of the floating cutting process was carried out in the rigid-flexible coupling numerical simulation model of root-cutting mechanism and garlic plant. The influence law of garlic conveying speed, extension spring preload force and stiffness on the floating displacement of the cutting component and the angular velocity of swing arm reset and its formation causes were analyzed by a single-factor simulation test. The key operating parameters of the root-cutting mechanism were optimized through the computerized virtual orthogonal test and fuzzy comprehensive evaluation.

**Results and discussion:**

The significance of the factors affecting the floating cutting performance decreased in the following order: extension spring preload force, garlic conveying speed and extension spring stiffness. The optimal parameter combination of the root cutting mechanism obtained from the optimization were as follow: extension spring preload force was 16 N, garlic conveying speed was 0.8 m/s, and extension spring stiffness was 215 N/m. Tests conducted with the optimal parameter combination yielded a root excision rate of 92.72%, which meets the requirements of Chinese garlic field harvesting quality. This study provides computer simulation optimization methods for the optimal design of the root-cutting mechanism, and also provides technical and equipment support for the full mechanization of garlic production in China.

## 1 Introduction

Garlic (*Allium sativum L*.) is an herb of the genus Allium in the lily family, whose bulbs have a high food value not only for direct consumption but also as a cooking ingredient or condiment for everyday dishes. According to the statistics of the Food and Agriculture Organization of the United Nations (FAO), China accounts for 80% of the global garlic production, while 90% of cultivated areas are located in Asia and Africa (FAOSTAT, 2020a; FAOSTAT, 2020b). China is the world’s largest garlic producer. Its perennial garlic planting area, harvest area, and export volume rank first in worldwide (FAOSTAT, 2020a; FAOSTAT, 2020b). **Figure 1** shows the garlic field production process, which has three major stages: sowing, field management and harvesting. In China, old machinery has been used for garlic sowing and field management, while harvesting is done manually or with small excavators. Highly efficient garlic combine harvesting equipment can be considered as “unavailable” (Yu et al., 2023). It is difficult to achieve combined harvesting of garlic in China due to the prevalence of mulching, narrow spaced dense planting and the tendency of garlic plants to fall over during harvest period. In 2022, the total mechanized harvesting area of garlic in China was less than 6%. The low level of harvest mechanization has hindered the development of China’s garlic industry. The slow development of combine harvesting technology is the main factor affecting the promotion and application of mechanized garlic harvesting technology in China.

**Figure 1:** Garlic field production process (sowing, field management, harvesting).

The garlic combine harvesting process includes garlic digging, soil removal, seedling cutting, root cutting, and bulb bagging (Zhao et al., 2020). Root-cutting is the most difficult process as well as the main factor that hiders the development of garlic combine harvesting technology (Yang et al., 2015; Quynh Anh et al., 2022). Owing to characteristics such as deep rooting, wide lateral growth of garlic roots, soft and tough roots, and the unsupported state of roots during cutting, it is difficult to efficiently remove the roots all at once. The size of the bulbs also varies, and traditional fixed cutters cannot be change according to the size of the bulb (Wang et al., 2018). Moreover, because the roots are attached to the root disc of the bulb, and when cutting the roots near the root disc, it is very easy to cause bulb cutting damage. It is a key technical challenge that must be addressed in the combine harvesting of garlic to achieve one-time and high-efficiency root removal without bulb damage.

To date, research on the root-cutting technology for garlic combine harvesting remains in the exploratory and experimental stages worldwide. Years of continuous and extensive literature searches have identified few academic reports on the mechanized garlic root-cutting technology. Yu et al. (2021b) developed a profiling, roller-type root-cutting mechanism for garlic combine harvesters. The rotational trajectory of the cutter was designed as a rotating hyperbolic surface that follows the shape of the lower surface of a garlic bulb. The operating parameters of the mechanism were determined, and the root fracture process was analyzed in detail by high-speed photographic tests. However, this mechanism was not highly adaptable to bulbs of different sizes. Cai (2019) developed a U-blade bite-type root-cutting mechanism for the primary processing of postharvest garlic, in which two symmetrically arranged special U-blades bite each other around their respective turning points to form a conical cutting track. By aligning the bottom of the bulb with the conical tip of the conical cutting track, both the garlic roots and root discs could be removed in one operation. However, this mechanism requires the manual orientation and placement of bulbs before cutting. Yang et al. (2022) proposed a noncontact positioning root-cutting method based on machine vision. They constructed a deep convolutional neural network with an improved YOLO v2 model to detect specific bulbs and roots, and predict the root-cutting line position. Two serrated disc cutters were automatically adjusted to the cutting line position for root-cutting. However, the complexity of the image acquisition environment requires improvements in image denoising technology. Using machine vision technology, Zhao et al. (2011) developed a special algorithm for the rapid positioning of the intersection of garlic bulb and roots. They used graphical user interface programming to develop an automatic and precise positioning system for the intersection of garlic bulb and roots, which provided a theoretical basis for the development and application of machine vision technology in an automated garlic root-cutting system. Thuyet et al. (2020) developed an automated grading and robotic-sorting system for root-trimmed garlic. The system used a deep convolutional neural network based image analysis technique to grade and sort root-trimmed garlic. This study provided a theoretical basis for the development and application of fully automated garlic root-cutting and bulb-sorting robots. The main garlic harvesting equipment being developed in China were garlic excavator and garlic seedling cutting combine harvester, while garlic combine harvesting equipment with root-cutting function is not yet available (Yu et al., 2021b). Erme (France), J.J. Broch (Spain) and Top Air (USA) are the main garlic harvesting equipment manufacturers in Europe and the United States. Their products include garlic excavators, garlic pickers, and stalk-cutting and baling-type garlic harvesters. However, these machines do not have a garlic root-cutting function. The HZ1 self-propelled garlic harvester by the Yanmar Company of Japan is the only garlic harvester with a root-cutting function from a developed country. The root-cutting mechanism consists of two superimposed serrated disc cutters. Because the serrated disc cutters are the fixed, the cutting height could not be adaptively adjusted according to the size of the bulb, resulting in poor root-cutting performance (Hou et al., 2021).

In recent years, the advances in computer simulation technology for agricultural machinery research have increased. The use of computer simulation technology has become an important step in the virtual simulation modeling and dynamic simulation analysis of crop mechanization harvesting to determine the interaction mechanism between harvesting machinery and crops, and to optimize the operating parameters. ADAMS is the most widely used software for the simulation and analysis of multibody system dynamics. Its rigid-flexible coupling modeling approach consists of three methods (Pu and Wu, 2009): the discrete beam method, modal neutral file (MNF) method, and AutoFlex method. The effects of the proposed method on crop-harvesting domains are discussed below. Using the discrete beam method, Wang et al. (2021) developed a flexible body model of the chrysanthemum stalk in ADAMS and fused it with a chrysanthemum picker to construct a rigid-flexible coupled numerical simulation model of the picker and chrysanthemum. The main factors affecting chrysanthemum picking were determined using dynamic simulation tests. Using the MNF method, Xie et al. (2020) completed the meshing of the sugarcane model in ANSYS, imported it into ADAMS, and fused it with the sugarcane top-breaking roller model to construct a rigid-flexible coupled numerical simulation model of the top-breaking rollers and sugarcane. The motion characteristics of sugarcane during top-breaking were studied using dynamic simulation tests. Shi et al. (2017) used the AutoFlex method to generate a flexible body model of the *Artemisia selengensis* (*A. selengensis*) stalk in ADAMS, which was fused with a cutter model of the *A. selengensis* harvester to construct a rigid-flexible coupled numerical simulation model of the cutter and *A. selengensis* stalk. Kinetic simulation analysis of the cutting process of the *A. selengensis* stalk was carried out, and the working parameters of the cutter were optimized by virtual simulation orthogonal tests. Yu et al. (2021a) used the AutoFlex method to transform a coffee stalk model into a flexible body in ADAMS, and constructed a simulation model of vibrating comb-type coffee threshing. The generalized force and sensor functions were used to monitor and control the shedding of coffee grains, and the dynamic simulation of the coffee threshing process was achieved. In addition, Chen et al. (2021) constructed finite element models of a garlic bulb and cutter based on ANSYS/LS-DYNA. Though the simulation analysis of root-disc cutting, they investigated the effects of the structural parameters of the cutter on the root-disc cutting force, and obtained the optimal structural parameters of the cutter. The abovementioned study serves as a reference of the present study in optimizing the floating root-cutting process of garlic using computer simulation technology.

To address the current problems of technological backwardness and poor operational quality of mechanized garlic root-cutting in China, this study combined the physical characteristics and agronomic requirements of garlic plants, and proposed an innovative floating root-cutting technology for garlic combine harvesters that enables the top alignment of bulb, adaptive profiling floating of cutter, and embedded cutting of roots. The kinematic and dynamic simulation analyses of the floating process of the root-cutting mechanism were conducted, and the optimal parameter combination of the root-cutting mechanism was obtained. The three main contributions of this study are as follows.

(1) The coordinate equations of the initial contact point of the bulb and a mathematical model of the floating displacement of the cutting component were established. The influence law and factors of the floating displacement of the cutting component in the two stages of floating were revealed. The theoretical basis for the optimal design of the root-cutting mechanism was provided.
(2) Using computer simulation techniques, the dynamic simulation analysis of the floating cutting process was conducted. The effects of each factor on the floating cutting performance were analyzed through single-factor simulation test. The key operating parameters of the root-cutting mechanism were optimized through virtual orthogonal test and fuzzy comprehensive evaluation. The computer simulation optimization method was provided for the optimal design of the root-cutting mechanism.
(3) Finally, the accuracy and reliability of the optimal parameter combination of the root-cutting mechanism were verified by simulation and field verification tests. The verification test results showed that the operating indexes of the root-cutting mechanism met the requirements of Chinese garlic field harvesting quality. The results of this study provide a reference for technological improvements and mechanism optimization of root-cutting for garlic combine harvesting in China.

## 2 Materials and methods

### 2.1 Structure of the root-cutting mechanism

The structure of the garlic root-cutting mechanism is shown in **Figure 2** and the root-cutting mechanism mainly consists of a clamping chain, alignment chain, roller brush, front rotary cutter, extension spring, swing arm, double elastic guide plates, and horizontal disc cutting component (hereinafter referred to as “cutting component”) (Yu et al., 2023). Among them, the clamping and alignment chains are in an inclined configuration. The double elastic guide plates were configured on both sides of the bulb running track and below the alignment chain. The double elastic guide plates with rubber pads were placed on the inside. The cutting component was configured below the double elastic guide plates, and is the main component for roots-bulb separation. It mainly consists of double protective fences, horizontal disc rotary cutter group, and DC motor. The double protective fences were arranged in parallel above the horizontal disc rotary cutter group. The exterior of the double protective fences could be fitted with rubber sleeves. One end of the swing arm was hinged to the frame, while the end was hinged to the cutting component. The two swing arms, cutting component and frame formed a parallel four-link structure. Therefore, during the floating cutting process, the cutting component moves in translation but did not rotate, thus ensuring that the spatial posture of the cutting component remained constant. The extension spring was connected to the frame at one end and to the swing arm at the other end; hence the cutting component produced elastic floating during the cutting process.

**Figure 2:** Structure of the root-cutting mechanism. 1. Clamping chain; 2. Alignment chain; 3. Double elastic guide plates; 4. Extension spring; 5. Double protective fences; 6. Horizontal disc rotary cutter group; 7. Horizontal disc cutting component; 8. Swing arm; 9. Front rotary cutter; 10. Roller brush.

### 2.2 Working principle of the root-cutting mechanism

The garlic plant enters the clamping chain from the clamping chain feed inlet. The clamping chain holds the upper stalk of the plant and transports it backward. Then, the lower stalk of the plant enters the alignment chain and the plant is transported backward by the clamping action of the clamping chain and the pushing action of the alignment chain. As the plant is transport backward, the high-speed rotating roller brush removes the soil that adhered to the roots and neatly combs the disorganized roots. The high-speed rotating front rotary cutter, which acts on the lower part of the roots, completes the pre-cutting of the roots and makes them form a neat cross-section. Owing to the inclined configuration of the clamping and the alignment chains (i.e., the distance between the fronts of the clamping and alignment chains was small, while the distance between their ends was large) and given that the alignment chains restrict the movement of the plant in the forward and backward directions, the bulb gradually approached the alignment chain and completed the top alignment. Once the bulb was firmly attached to the alignment chain, it restricted the movement of the plant in both upward and downward directions. As the distance between the clamping and alignment chains increased, the bulb slid downward relative to the clamping chain; however, it always remained close to the alignment chain and was transported backward. Subsequently, the double elastic plates guided the bulb into the cutting channel to prevent its lateral deflection. The lower surface of the bulb was pressed against the double protective fences, which brought the cutting component close to it. The roots were simultaneously cut off by the horizontal disc rotary cutter group through the double protective fences, thus separating the roots from the bulb.

### 2.3 Kinematic analysis of the floating process of the root-cutting mechanism

The elastic floating of cutting component is an important guarantee for efficient and low damage cutting of the roots. Studying the kinematic characteristics of elastic floating of the cutting component provides a theoretical basis for optimizing the root-cutting mechanism.

From a kinematic perspective, the floating displacement of the cutting component and the position of the initial contact point between the bulb and cutting component are the key parameters reflecting the kinematic characteristics of the elastic floating of the cutting component (Yu et al., 2021c). Because the floating displacement of the cutting component determines the relative position of the bulb and the cutting component, it can be used to determine the distance between the rotary cutter group and root disc during the floating process. Simultaneously, the floating displacement of the cutting component determines the elongation of the extension spring, which affects the squeezing force applied to the lower surface of the bulb. The position of the initial contact point between the bulb and cutting component (hereinafter referred to as the initial contact point of the bulb) determines the floating displacement of the cutting component in two different floating phases and the point where the bulb is subjected to the maximum impact force.

In this section, the mathematical model of the floating displacement of the cutting component and the coordinate equations of the initial contact point of the bulb are established through theoretical analysis. The purpose is to clarify the influence law and factors of the floating displacement of the cutting component and the initial contact point of the bulb.

#### 2.3.1 Determination of the initial contact point of the bulb

As shown in **Figure 3**, the hinge point of lower swing arm *o* is the origin of the coordinates, the conveying direction of the alignment chain is the positive direction along the *x*-axis, while the upward direction is the positive direction along *y*-axis. The bulb is considered an ellipsoid, with a long axis (bulb diameter) of 2*a* and short axis (bulb height) of 2*b*. The equation of the bulb elliptical outline at the initial moment of contact between the bulb and cutting component is expressed as:

**Figure 3:** Schematic diagram of the relative position of the floating process of the cutting component.


(1) $$\frac{{\left(x-x_{o^{\prime }}\right)}^{2}}{a^{2}}+\frac{{\left(y-y_{o^{\prime }}\right)}^{2}}{b^{2}}=1$$

where, *x*_o′_ and *y*_o′_ are the horizontal and vertical coordinates of the center point *o*′ of the bulb (m).

As seen from **Figure 2**, the protective fence has two vertical edges at the front and back, a top beveled edge, and a top horizontal edge. The top beveled edge is the part that makes initial contact with the bulb and guides it to the top horizontal edge. As shown in **Figure 3**, a line *mn*, which coincides with the top beveled edge of the protective fence, was created. The slope *k* of the line *mn* remained constant during the floating process. At the initial moment of contact between the bulb and cutting component, the equation of line *mn* is expressed as:


(2) y=kx+c

where, *k* is the slope of line *mn* and *c* is the value of the vertical coordinate of the intersection at the line *mn* and *y*-axis.

As seen from **Figure 3**, the tangent point between line *mn* and the bulb elliptical outline is the initial contact point *i* of the bulb. From Equations (1) and (2), the coordinates of the initial contact point *i* of the bulb are expressed as:


(3) $$\left\{ \begin{array}{c} x_{i}=\frac{a^{2}k}{\sqrt{a^{2}k^{2}+b^{2}}}+x_{o^{\prime }}\\ y_{i}=-\frac{b^{2}}{\sqrt{a^{2}k^{2}+b^{2}}}+y_{o^{\prime }} \end{array}\right.$$

where, *x_i_* and *y_i_* are horizontal and vertical coordinates of the initial contact point *i* of the bulb (m). As seen from Equation (3), the position of the initial contact point of the bulb is related to the size of the elliptical outline of the bulb, the coordinates of the center point of the bulb, and the slope of the top beveled edge of the protective fence. To reduce the bulb collision damage, the position of the initial contact point of the bulb should be shifted toward the bottom of the bulb during the cutting process.

#### 2.3.2 Mathematical model of the floating displacement of the cutting component

After the bulb made contact with the top beveled edge of the protective fence, the plant continued to be transported backward, the bulb was pressed against the double protective fences to float the cutting component downward. In this study, the downward floating process of the cutting component was divided into two stages. In the first stage, the bulb makes contact with the top beveled edge of the protective fence, and the cutting component floats downward. In the second stage, the bulb makes contact with the top horizontal edge of the protective fence, and the cutting component floats downward.

In the first stage, relative sliding between the bulb and protective fence occurred. The points of action of the squeezing and frictional forces exerted by the top beveled edge of the protective fence on the bulb remained the same. From the positional relationship shown in **Figure 3**, the floating displacement *l*_1_ of the cutting component in the first stage of floating is expressed as:


(4) $$l_{1}=\left|H_{2}-y_{i}\right|=\left|\frac{b^{2}}{\sqrt{a^{2}k^{2}+b^{2}}}+\left(H_{2}-y_{o^{\prime }}\right)\right|$$

where, *H*_2_ is the initial height of the top horizontal edge of the protective fence (m). In the mechanism design, when the slope of the top beveled edge of the protective fence was determined, the initial height *H*_2_ should be greater than the height *y_i_* of the initial contact point of the bulb to minimize the bulb collision damage. Otherwise, the bulb will collide with the bending area between the top beveled edge and top horizontal edge of the protective fence, which could damage the bulb. As seen from Equation (4), the first stage floating displacement *l*_1_ was positively correlated with the bulb height 2*b* and initial height *H*_2_, and negatively correlated with the bulb diameter 2*a* and the slope of the top beveled edge of the protective fence.

When the height of the top horizontal edge of the protective fence was gradually lowered and below the initial contact point *i* of the bulb, it meant the second stage of floating. The bulb disengaged from the top beveled edge and made contact with the top horizontal edge of the protective fence. The bulb was pressed against the top horizontal edge of the protective fence, which caused the cutting component to continue floating downward. The point of action of the squeezing and frictional forces exerted by the top horizontal edge of the protective fence on the bulb gradually lowered. When the lower surface of the bulb was above the horizontal edge of the protective fence, the squeezing and frictional forces on the bulb shifted toward the lowest point at the bottom of the bulb, and the cutting component floated downward to the lowest point. At this time, the floating displacement *l*_2_ of the cutting component increased to the maximum value expressed as:


(5) $$l_{2}=\left|y_{i}-y_{o^{\prime }}+b\right|=\left|b-\frac{b^{2}}{\sqrt{a^{2}k^{2}+b^{2}}}\right|$$

As seen from Equation (5), the floating displacement *l*_2_ of the cutting component in the second stage of floating is related to the bulb diameter 2*a*, bulb height 2*b*, and slope *k* of the top beveled edge of the protective fence. As the point of action of squeezing and frictional forces exerted by the top horizontal edge of the protective fence on the bulb gradually lowered, the change of the point of action causes the change of the damaged part of the bulb and thus expanded the damaged area of the bulb. The larger the floating displacement *l*_2_ of the cutting component, the wider the damaged area of the bulb would be, and the long the time of the squeezing and frictional forces on the bulb would be.

The above analysis not only obtained the coordinate equations of the initial contact point between the bulb and cutting component and the mathematical model of the floating displacement of the cutting component, but also revealed the influence law and factors of the floating displacement of the cutting component in the two stages of floating. These provide a theoretical reference for the analysis of bulb collision damage, extension spring elongation and preload force, and kinematic analysis of the elastic floating of the cutting component.

### 2.4 Numerical simulation modeling

ADAMS is a multi-body system dynamics analysis software that can simulate the floating cutting process of the root-cutting mechanism to significantly reduce the development cost and cycle time of the mechanism (Wang et al., 2022). This section used the ADAMS software to carry out the dynamic simulation of the floating cutting process of the root-cutting mechanism, with the aim of studying the effects of different operating parameters on the floating cutting performance to optimize the parameters of the root-cutting mechanism.

#### 2.4.1 Models of garlic plant and root-cutting mechanism

**Figure 4** shows the parts of a garlic plant, which include the stalk, bulb, and roots. As shown in **Figure 5**, the ANSYS and ADAMS coupling method was used to establish the flexible body model of the stalk and bulb (Yu et al., 2023). First, the 3D models of the stalk and bulb were imported into the Mechanical APDL module in ANSYS for meshing. Then, the modal neutral files of the stalk and bulb were imported into ADAMS using the coupling interface “ADAMS Flex: Create a Flexible Body”. Finally, the model properties and modalities of each order were checked and verified. Jinxiang garlic is a typical garlic variety grown in China′s main garlic producing areas. Flexible body model of stalk with a diameter of 13 mm and a length of 230 mm was constructed and a flexible body model of bulb with a diameter of 61 mm and a height of 45 mm was constructed. The densities of the stalk and bulb were 855.2 kg/m^3^ and 1057 kg/m^3^; the Poisson′s ratios were 0.30 and 0.23; and the elastic modulus were 8.0×10^6^ Pa and 2.38×10^7^ Pa, respectively.

**Figure 4:** The composition of garlic plant.

**Figure 5:** The flexible body model of the garlic plant.

As shown in **Figure 5**, the ADAMS discrete beam method was used to construct a flexible body model for the garlic root group (Yu et al., 2023). First, a 3D model of the root group was created and then imported into ADAMS to discretize the single root one by one. The diameter and length of a single root were 1.6 mm and 63 mm; the density, Poisson′s ratio, and elastic modulus of the root were 837.3 kg/m^3^, 0.385, and 2.26×10^6^ Pa, respectively. A single root was discretized into flexible beams.

A flexible body model of the garlic plant was constructed by fusing the stem, bulb and root group.

Model of root-cutting mechanism: A 3D simplified model ofv the main components of the root-cutting mechanism was created by INVENTOR, and then imported into ADAMS along with the material properties of each component (Wang et al., 2013).

#### 2.4.2 Rigid-flexible coupling model of the root-cutting mechanism and garlic plant

As shown in **Figure 6**, based on the kinematic analysis of the root-cutting mechanism, constraints, forces, drives, and dummy objects were added to build a rigid-flexible coupling model of the root-cutting mechanism and garlic plant in ADAMS (Yu et al., 2023). The stationary components were fixed to the reference system, while the revolute and translational pairs were used to define the constraints between components with rotational and linear relative motion relationships (Prastiyo and Fiebig, 2021). Simultaneously, dummy objects were constructed to assist the addition of motion constraints between the flexible body model of the garlic plant and interacting components. Contact constraints between the flexible body model of garlic plant and the interacting components were applied.

**Figure 6:** Rigid-flexible coupling model of the root-cutting mechanism and garlic plant.

The impact function (IMPACT) was used to define the contact force between the bulb and protective fence, which has a contact type of Flex Body to Solid. The general expression of the impact function (Chen and Dun, 2012; Xie, 2019), which consists of the elastic force generated by the mutual extrusion of two objects and the damping force generated by their relative motion, is expressed as:


(6) $$Q_{Impact}\left(x_{i}\right)=\left\{ \begin{array}{l} 0\;x_{i}<x_{0}\\ k_{\text{s}}{\left(x_{0}-x_{i}\right)}^{e}-step\left(x_{i},x_{0}-d,1,x_{0},0\right)\cdot c_{\max}\;x_{i}\geq x_{0} \end{array}\right.$$

where, Q*_Impact_* is the contact force between two objects (N); *x_i_* is the actual distance of the collision zone of two objects (mm); *x*_0_ is the initial distance of the collision zone before the contact between two objects (mm); *e* is the contact force index; *d* is the penetration depth (mm); *c*_max_ is the maximum damping coefficient (N·s/mm^-1^); *step* is the step function that prevents the discontinuity of damping force during the collision; and *k_s_* is the contact stiffness coefficient (N/mm). The Hertz collision contact model was used to calculate the contact stiffness coefficient *k_s,_* which is expressed as:


(7) $$k_{s}=\frac{16R^{*}E^{*}{\;}^{2}}{9}$$

where, R^*^ is the equivalent relative radius of curvature (mm); $\frac{1}{R^{*}}=\frac{1}{R_{1}}+\frac{1}{R_{2}}$ , where *R*_1_ and *R*_2_ are the radius of curvature of the bulb (17.25 mm) and protective fence (1.5 mm) in the collision zone; E^*^ is the equivalent elastic modulus (Mpa); $\frac{1}{E^{*}}=\frac{1-\mu_{1}{\;}^{2}}{E_{1}}+\frac{1-\mu_{2}{\;}^{2}}{E_{2}}$ , where *E*_1_ and *E*_2_ are the elastic moduli of the bulb and protective fence, respectively. The elastic modulus of the protective fence is 2.1×10^5^ MPa; *μ*_1_ and *μ*_2_ are the Poisson’s ratios of the bulb and protective fence, respectively. The Poisson′s ratio of the protective fence is 0.3. According to Equation (7), the contact stiffness coefficient *k_s_* between the bulb and protective fence is 1546 N/mm. The parameters of the impact function are listed in **Table 1**. (The parameters taken from reference (Chen and Dun, 2012) or the official recommended values of ADAMS software were tested and modified).

**Table 1:** The parameters of the impact function.

Parameters	Values
Contact Stiffness Coefficient *k_s_* (N·mm^-1^)	1546
Contact Force Index *e*	2.2
Damping Coefficient *c*_max_ (N·s·mm^-1^)	10
Penetration Depth *d* (mm)	0.1

The drive was added to the clamping chain, alignment chain, and rotary cutter group. To reduce the residual root length after cutting, the root disc should be parallel to the rotary plane of the rotary cutter group when it cuts the roots. The above requirements could be achieved by the reasonable configuration of the speed ratio of the alignment and clamping chains. According to the research method of Yu et al. (2021b), the speed ratio between the alignment and the clamping chains was calculated as 1.015 based on the displacements of the alignment and the clamping chains when the garlic plant was jointly clamped and transported.

## 3 Dynamic simulation of the floating cutting process

The elastic expansion and contraction of the extension spring made the root-cutting mechanism drive the up and down floating of the cutting component. By optimizing the mechanical structure, motion parameters, and mechanical parameters of the extension spring, it would be possible to achieve the protection fence always closed to the lower bulb surface during the floating cutting process. After the basic structural form and parameters of the root-cutting mechanism were determined, the optimal floating cutting performance of the root-cutting mechanism can be achieved by optimizing the motion parameters of the root-cutting mechanism and the mechanical parameters of the extension spring.

In this section, using computer simulation techniques, the dynamic simulation study of the floating cutting process would be carried out in the rigid-flexible coupling numerical simulation model of root-cutting mechanism and garlic plant. Firstly, through single-factor simulation test, the influence law of the motion parameters of the root-cutting mechanism and the mechanical parameters of the extension spring on the floating cutting performance and its formation causes would be analyzed. Then, through virtual orthogonal test and fuzzy comprehensive evaluation, the optimal parameter combination of the root-cutting mechanism would be determined and verification test would be carried out.

### 3.1 Single-factor simulation test

#### 3.1.1 Test index

The root excision rate is the main index used to evaluate the quality of garlic root-cutting. The key to the efficient cutting of garlic roots is to ensure that the protective fence is always close to the lower surface of the bulb during the floating cutting process. Because the rotary cutter group was positioned beneath the protective fence, and the cutting edge was close to the protective fence, the protective fence was close to the lower surface of the bulb, which ensured that the cutting edge was close to the root disc when cutting the root, and only a short length of the root remained after cutting.

The above theoretical analysis and preliminary experimental study showed that two main technical problems must be solved to ensure that the protective fence is always close to the lower surface of the bulb. First, when the bulb collides with the cutting component, the cutting component is ejected downward by the contact force and temporarily moves away from the lower surface of the bulb, making it impossible for the protective fence to be close to the lower surface of the bulb in the early stage of cutting. Second, after the completion of floating cutting process (i.e., the garlic is disengaged from the cutting component), it takes time for the cutting component to rise from the lowest point to the highest point of floating. Thus, when the next garlic enters the protective fence, the protective fence has yet to return to the highest point. This will affect the subsequent garlic to repeat the floating cutting operation successively. To quantitatively assess the floating cutting performance of the root-cutting mechanism, the floating displacement of the cutting component and angular velocity of swing arm reset (i.e., the angular velocity of the swing arm when the bulb disengaged from the cutting component and the cutting component floated upward) were used as the single-factor simulation test indexes.

#### 3.1.2 Test factor

Based on kinematic analysis results of the floating process of the root-cutting mechanism and the pre-test results of the simulation, this study selected the key factors affecting the floating cutting performance, such as the extension spring preload force, extension spring stiffness, and garlic conveying speed (i.e., clamping chain conveying speed) as the test factors to carry out the simulation analysis, and devoted to investigate the influence law of each factor on the floating cutting performance and its formation causes. The pre-test results of the extension spring preload force showed that to reduce the effects of collisions on the downward floating of the cutting component, the minimum preload force of 12 N was taken. The maximum preload force of 16 N was chosen to reduce the bulb collision damage caused by excessive preload force. Therefore, the extension spring preload forces were set as 12, 13, 14, 15 and 16 N. If the extension spring stiffness or preload force was different, the tension required to stretch the spring was different, then there may be an effect on the floating effect of the cutting component. To study the effects of the spring stiffness on the floating process, the test began with the minimum value of 15 N/m. Based on the results of the preliminary bench test, the selected extensile spring stiffness values were 15, 65, 115, 165 and 215 N/m. If garlic conveying speed was different, impact force between the bulb and the protective fence was different, then there may be an effect on the floating effect of the cutting component. The selected garlic conveying speeds were 0.8, 0.9, 1.0, 1.1 and 1.2 m/s.

#### 3.1.3 Single-factor test results and analysis

(1) Effect of extension spring preload force on the floating cutting performance

In the single-factor test of the extension spring preload force, the garlic conveying speed and extension spring stiffness were set as 0.8 m/s and 215 N/m, respectively. The effect of the extension spring preload force on the floating displacement of the cutting component and angular velocity of swing arm reset was obtained through the simulation test, as shown in **Figure 7**. First, the changing process of the floating displacement of the cutting component during the simulation was analyzed, as shown in **Figure 7A**. When the simulation started, the displacement of the cutting component first remained constant. When the bulb collided with the top beveled edge of the protective fence, the cutting component was ejected and displaced downward. Then, the ejected cutting component gradually rose under the action of the extension spring. After the top horizontal edge of the protective fence made contact with the lower surface of the bulb and was pressed against it, and the displacement of the cutting component remained constant. When the root-cutting operation was completed, the bulb disengaged from the cutting component and the cutting component floated upward again. Finally, the cutting component returned to the height before the collision. The displacement of the cutting component remained constant while waiting for the subsequent garlic to repeat the operation.

**Figure 7:** Effects of the extension spring preload force on the floating displacement of the cutting component and the angular velocity of swing arm reset. In **(A)**, the red circle marked the downward displacement caused by the cutting component being ejected downward; In **(B)**, the red circle marked the change in the angular velocity of swing arm during the reset phase of the cutting component.

In **Figure 7A**, the red circle marked the downward displacement caused by the cutting component being ejected downward. As seen from **Figure 7A**, the greater the preload force, the smaller the downward displacement caused by the cutting component being ejected downward would be, and the smaller the floating displacement of the cutting component would be. The possible reasons are as follows. The greater the preload force, the greater the resistance of the downward floating of the cutting component would be, the smaller the initial speed of the cutting component caused by the bulb collision would be, thus decreasing the floating displacement of the cutting component.

When the root-cutting operation was completed, the bulb gradually disengaged from the cutting component; under the action of the extension spring, the cutting component gradually floated upward with a certain reset angular velocity. At this time, the angular velocity of swing arm reset determined the time of the cutting component reset, which affected the repeated cutting operation of the subsequent garlic. In **Figure 7B**, the red circle marked the change in the angular velocity of swing arm during the reset phase of the cutting component, i.e., the change in the angular velocity of swing arm reset. As shown in **Figure 7B**, the angular velocity of swing arm reset increased with the increase of the extension spring preload force. The possible reasons are as follows. The greater the preload force, the greater the tension of the extension spring on swing arm would be, and the higher the angular acceleration of swing arm reset would be, thus increasing the angular velocity of swing arm reset.

(2) Effect of extension spring stiffness on the floating cutting performance

In the single-factor test of the extension spring stiffness, the extension spring preload force and garlic conveying speed were set as 16 N and 0.8 m/s, respectively.

The effects of the extension spring stiffness on the floating displacement of the cutting component are shown in **Figure 8A**. The floating displacement of the cutting component decreased with the increase of the extension spring stiffness, but this trend was not obvious. The possible reasons are as follows. The greater the stiffness, the greater the tension required for the extension spring to elongate the same length would be, the greater the resistance of the floating downward of the cutting component would be, and the smaller the initial speed of the cutting component caused by the bulb collision would be, thus decreasing the floating displacement of the cutting component. When the stiffness increased to a certain value, the floating displacement of the cutting component was smaller, and the variation of the floating displacement of the cutting component caused by different stiffness was not obvious.

**Figure 8:** Effects of the extension spring stiffness on the floating displacement of the cutting component and the angular velocity of swing arm reset. In **(A)**, the red circle marked the downward displacement caused by the cutting component being ejected downward; In **(B)**, the red circle marked the change in the angular velocity of swing arm during the reset phase of the cutting component”.

The effects of the extension spring stiffness on the angular velocity of swing arm reset are shown in **Figure 8B**. The angular velocity of swing arm reset was basically constant with the increase of the extension spring stiffness. The possible reasons are as follows. The five extension spring stiffnesses tested in the single-factor test corresponded to the five tensions of the extension spring. However, when the bulb disengaged from the cutting component and the cutting component gradually floated upward, compared with the gravity of the cutting component, the five tensions of the extension spring did not differ much. So the five angular accelerations of swing arm reset caused by five tensions of the extension spring did not differ much, thus leading to little change in the angular velocity of swing arm reset.

(3) Effect of garlic conveying speed on the floating cutting performance

In the single-factor test of the garlic conveying speed, the extension spring stiffness and extension spring preload force were set as 215 N/m and 16 N, respectively.

The effects of the garlic conveying speed on the floating displacement of the cutting component are shown in **Figure 9A**. The floating displacement of the cutting component increased with the increase of the garlic conveying speed. The possible reasons are as follows. Because the cutting component was connected to the frame by an extension spring, at the moment of collision between the bulb and the cutting component, it is approximated as an elastic collision. According to the laws of conservation of momentum and conservation of energy, the higher the garlic conveying speed, the greater the speed of the cutting component after the collision would be, thus increasing the floating displacement of the cutting component.

**Figure 9:** Effects of the garlic conveying speed on the floating displacement of the cutting component and the angular velocity of swing arm reset. In **(A)**, the red circle marked the downward displacement caused by the cutting component being ejected downward; In **(B)**, the red circle marked the change in the angular velocity of swing arm during the reset phase of the cutting component”.

The effects of the garlic conveying speed on the angular velocity of swing arm reset are shown in **Figure 9B**. The angular velocity of swing arm reset was basically constant with the increase of the garlic conveying speed. The possible reasons are as follows. As shown in **Figure 9A**, the displacement curve of the cutting component was already in the horizontal state before the bulb disengaged from the cutting component, which means that the protective fence was already close to the lower surface of the bulb. Therefore, for the five states of garlic conveying speed, the cutting component was at the same displacement and was subject to the same tension of the extension spring when the bulb disengaged from the cutting component. Thus, the angular velocity of swing arm reset was the same.

### 3.2 Virtual orthogonal test

Through above-mentioned single-factor simulation test, the influence law of the motion parameters of the root-cutting mechanism and the mechanical parameters of the extension spring on the floating cutting performance and its formation causes were investigated. In order to select the parameter combination that were as optimal as possible for the floating displacement of the cutting component and the angular velocity of swing arm reset, and further investigate the combined effects of extension spring preload force *A*, extension spring stiffness *B*, and garlic conveying speed *C* on the floating cutting performance, a three-factor, three-level virtual orthogonal test would be conducted in this section.

#### 3.2.1 Design and scheme of virtual orthogonal test

To facilitate the quantitative assessment, the maximum floating displacement *l* of the cutting component at the moment of collision between the bulb and cutting component, and the maximum angular velocity *ω* of swing arm reset at the moment the bulb disengaged from the cutting component were selected as the quantitative assessment indexes of the virtual orthogonal test. The maximum floating displacement *l* of the cutting component is the increase of the displacement of the cutting component before the collision and the maximum displacement of the cutting component after the collision. Both indexes were automatically obtained by the ADAMS/postprocessor module. According to the above single-factor test results, the extensile spring preload force was selected as 14, 15, and 16 N, the extensile spring stiffness was 115, 165, and 215 N/m, and the conveying speed was 0.8, 0.9, and 1.0 m/s. The test was designed using the L_9_(3^4^) orthogonal test table. The test scheme is presented in **Table 2**.

**Table 2:** Test schemes and results of virtual orthogonal tests.

Test Number	Extension Spring Preload Force *A*		Extension Spring Stiffness *B*	Garlic Conveying Speed *C*	Maximum Floating Displacement of The Cutting Component *l* (mm)	Maximum Angular Velocity of Swing Arm Reset *ω* (deg·s^-1^)
1	1(14)		1(115)	1(0.8)	4.45	45.50
2	1(14)		2(165)	2(0.9)	5.16	46.49
3	1(14)		3(215)	3(1.0)	5.90	47.13
4	2(15)		1(115)	2(0.9)	4.78	52.01
5	2(15)		2(165)	3(1.0)	5.45	52.06
6	2(15)		3(215)	1(0.8)	4.03	52.94
7	3(16)		1(115)	3(1.0)	5.15	56.43
8	3(16)		2(165)	1(0.8)	3.81	57.29
9	3(16)		3(215)	2(0.9)	4.39	58.58
Maximum Floating Displacement of The Cutting Component *l*	*K*_11_	15.51	14.38	12.29		
	*K*_12_	14.26	14.42	14.33		
	*K*_13_	13.35	14.32	16.5		
	Range	2.16	0.10	4.21		
	Significance Sequence of Factors *C>A>B* Optimal Parameter Combination *C_1_A_3_B_3_*					
Maximum Angular Velocity of Swing Arm Reset *ω*	*K*_21_	139.12	153.94	155.73		
	*K*_22_	157.01	155.84	157.08		
	*K*_23_	172.3	158.65	155.62		
	Range	33.18	4.71	1.46		
	Significance Sequence of Factors *A>B>C* Optimal Parameter Combination *A_3_B_3_C_2_*					

K_11_~K_13_ were the sum of the maximum floating displacement of the cutting component measured for a factor at level 1, level 2 and level 3, respectively; K_21_~K_23_ were the sum of the maximum angular velocity of swing arm reset measured for a factor at level 1, level 2 and level 3, respectively.

#### 3.2.2 Orthogonal test results and analysis

Based on the experimental scheme above, virtual orthogonal simulation tests were conducted, and the test results are listed in **Table 2**. Using IBM SPSS Statistics 22 software, the data processing and statistical analysis of the test results were performed (Gong et al., 2012; Li and Zhang, 2015).

First, range analysis was conducted on the test results. The range analysis results are listed in **Table 2**. The significance of the factors affecting the maximum floating displacement of the cutting component decreased in the following order: garlic conveying speed, extension spring preload force, and extension spring stiffness. The optimal parameter combination was *C*_1_ *A*_3_ *B*_3_; The significance of the factors affecting the maximum angular velocity of swing arm reset decreased in the following order: extension spring preload force, extension spring stiffness, and garlic conveying speed. The optimal parameter combination was *A*_3_ *B*_3_ *C*_2_.

Second, ANOVA was performed on the test results. The ANOVA results are summarized in **Table 3**. The degree of influence of factors on the maximum floating displacement of the cutting component and the maximum angular velocity of swing arm reset varied. At the 95% confidence level, the effects of the garlic conveying speed and extension spring preload force on the maximum floating displacement were highly significant (*P*< 0.01), and the effects of extension spring stiffness on the maximum floating displacement were not significant (*P* > 0.05). At the 95% confidence level, the effects of the extension spring preload force on the maximum angular velocity were highly significant (*P*< 0.01), the effects of extension spring stiffness on the maximum angular velocity was significant (0.01< *P*< 0.05) and the effects of garlic conveying speed on the maximum angular velocity were not significant (*P* > 0.05).

**Table 3:** ANOVA of virtual orthogonal tests.

Item	Source	Sum of Squares	D*f*	Mean Squares	*F* Value	*P* Value
Maximum Floating Displacement of The Cutting Component *l*	*A*	0.784	2	0.392	108.557	0.0091
	*B*	0.002	2	0.001	0.234	0.8105
	*C*	2.955	2	1.477	409.148	0.0024
	Error	0.007	2	0.004		
Maximum Angular Velocity of Swing Arm Reset *ω*	*A*	183.861	2	91.930	3395.053	0.0003
	*B*	3.743	2	1.872	69.122	0.0143
	*C*	0.441	2	0.220	8.137	0.1094
	Error	0.054	2	0.027		

P<0.01 (Highly significant), 0.01<P<0.05 (Significant), P>0.05 (Not significant).

#### 3.2.3 Fuzzy comprehensive evaluation and comprehensive optimization

The above analysis revealed that the three factors (i.e., such as extension spring preload force, extension spring stiffness, and garlic conveying speed) had different orders of significance, different significance, and different optimal parameter combinations for the maximum floating displacement of the cutting component and maximum angular velocity of swing arm reset. In view of this, it is necessary to conduct a comprehensive evaluation of the two indexes obtained from each group of tests. Based on the comprehensive evaluation results of floating cutting performance for each group test, the comprehensive optimization of factors was carried out to obtain the parameter combination that were as optimal as possible for the floating displacement of the cutting component and the angular velocity of swing arm reset.

Owing to orders of magnitude and dimensions of the two indexes were different, the fuzzy comprehensive evaluation method (Xu et al., 2021) was used to establish the membership model of the two indexes and obtain the same orders of magnitude and dimensionless membership values. The maximum floating displacement of the cutting component was a small offset index, i.e., the smaller the maximum floating displacement, the better. Its membership model is shown in Equation (8). The maximum angular velocity of swing arm reset was a large offset index, i.e., the larger the maximum angular velocity, the better. Its membership model is shown in Equation (9).


(8) $$t_{1n}=\frac{l_{\max}-l_{n}}{l_{\max}-l_{\min}}\left(n=1,2,\ldots .9\right)$$

(9) $$t_{2n}=\frac{\omega_{n}-\omega_{\min}}{\omega_{\max}-\omega_{\min}}\left(n=1,2,\ldots .9\right)$$

where *t*_1_ *_n_* and *t*_2_ *_n_* are the membership values of the maximum floating displacement *l* of the cutting component and the maximum angular velocity *ω* of swing arm reset for the *n*th test, respectively; *l*_max_ and *l*_min_ are the maximum and minimum values of index *l*; *l_n_* is the value of index *l* for the *n*th test; *ω*_max_ and *ω*_min_ are the maximum and minimum values of index *ω*; *ω_n_* is the value of index *ω* for the *n*th test; *n* is the test number. The membership values *t*_1_ *_n_* and *t*_2_ *_n_* were obtained from Equations (8) and (9), respectively, and are listed in **Table 4**.

**Table 4:** Comprehensive scores of the two indexes.

Test Number	Membership values of the maximum floating displacement of the cutting component *t*_1_ *_n_*	Membership values of the maximum angular velocity of swing arm reset *t*_2_ *_n_*	Comprehensive scores *U*
1	0.694	0	0.416
2	0.354	0.076	0.243
3	0	0.125	0.050
4	0.536	0.498	0.521
5	0.215	0.502	0.330
6	0.895	0.569	0.765
7	0.359	0.836	0.550
8	1	0.901	0.960
9	0.722	1	0.833

The fuzzy relationship matrix ***T_n_*** was constructed from the membership values of the two indexes. The fuzzy relationship matrix ***T_n_*** is expressed as:


(10) $$T_{n}=\left(\begin{array}{ccc} t_{11} & \cdots & t_{19}\\ \vdots & \ddots & \vdots \\ t_{21} & \cdots & t_{29} \end{array}\right)$$

This test was dedicated to reducing the maximum floating displacement of the cutting component and the maximum angular velocity of swing arm reset. According to the importance of the two indexes, the weight of the maximum floating displacement of the cutting component was set as 0.6 and the weight of the maximum angular velocity of swing arm reset was set as 0.4. Thus, the weight assignment set ***W*** was constructed as ***W*** = [0.6 0.4].

According to the fuzzy relationship matrix ***T_n_*** and the weight assignment set ***W***, the comprehensive score set ***U*** was obtained by fuzzy transformation, where ***U*** =*W*·*T_n_*. The comprehensive scores of floating cutting performance for each test were obtained, as listed in **Table 4**. The higher the comprehensive score, the better the performance of the test scheme would be.

In this study, the comprehensive scores of floating cutting performance were used as the comprehensive optimization basis of the root-cutting mechanism. The Shapiro-Wilk test was conducted using the IBM SPSS Statistics 22 software for comprehensive scores of floating cutting performance of the root-cutting mechanism in **Table 4**. The *P* value of the Shapiro-Wilk test was 0.957 (*P* > 0.05). The results indicate that the comprehensive scores of floating cutting performance of the root-cutting mechanism obtained from nine groups of simulation tests conformed to a normal distribution. Range analysis was performed on the comprehensive scores. From the range analysis results in **Table 5**, it could be seen that the significance of the factors affecting the floating cutting performance decreased in the following order: extension spring preload force, garlic conveying speed, and extension spring stiffness. The optimal parameter combination was *A*_3_ *C*_1_ *B*_3_ (i.e., extension spring preload force of 16 N, garlic conveying speed of 0.8 m/s, and extension spring stiffness of 215 N/m). Based on the range analysis results, a radar diagram that was drawn to visually describe the effects of factors on the comprehensive scores is shown in **Figure 10**. As seen from **Figure 10**, the comprehensive score is positively correlated with the extension spring preload force and stiffness and negatively correlated with the garlic conveying speed. ANOVA was performed on the comprehensive scores. The ANOVA results are shown in **Table 6**, which revealed that the effects of the extension spring preload force and garlic conveying speed on the comprehensive score were highly significant (*P*< 0.01), while the effect of extension spring stiffness on the comprehensive score was not significant (*P* > 0.05) at the 95% confidence level.

**Table 5:** Range analysis of comprehensive scores.

Item	Extension Spring Preload Force *A*	Extension Spring Stiffness *B*	Garlic Conveying Speed *C*
*K*_31_	0.709	1.487	2.141
*K*_32_	1.616	1.533	1.597
*K*_33_	2.343	1.648	0.930
Range	1.634	0.161	1.211
Significance Sequence of Factors *A*>*C*>B			
Optimal Parameter Combination *A*_3_ *C*_1_ *B*_3_			

K_31_~K_33_ were the sum of the comprehensive scores for a factor at level 1, level 2 and level 3, respectively.

**Figure 10:** Effects of factors on the comprehensive scores for the floating cutting performance. Note: *A*_1_ *~A*_3_ are the level 1, level 2 and level 3 of the extension spring preload force, respectively; *B*_1_ *~B*_3_ are the level 1, level 2 and level 3 of the extension spring stiffness, respectively; *C*_1_ *~C*_3_ are the level 1, level 2 and level 3 of the garlic conveying speed, respectively; The nine radial axes in the figure are the comprehensive scores for the floating cutting performance.

**Table 6:** ANOVA of comprehensive scores.

Source	Sum of Squares	D*f*	Mean Squares	*F* Value	*P* Value
Extension Spring Preload Force *A*	0.447	2	0.223	1301.815	0.0009
Extension Spring Stiffness *B*	0.005	2	0.002	12.873	0.0777
Garlic Conveying Speed *C*	0.245	2	0.123	716.903	0.0016
Error	0.0004	2	0.0002		

#### 3.2.4 Simulation verification of optimization results

In order to verify the accuracy and reliability of the above optimization results, we needed to measure the performance of the optimal parameter combination through simulation test. The simulation verification test was conducted in the rigid-flexible coupling model of the root-cutting mechanism and garlic plant constructed in section 2.4. Same as the above virtual orthogonal test, the simulation model used the impact function method (IMPACT) to define the contact force between the bulb and protective fence, its contact type was Flex Body to Solid, the contact stiffness coefficient was 1546 N/mm, the contact force index was 2.2, the damping coefficient was 10 N·s/mm, the penetration depth was 0.1 mm, and the speed ratio between the alignment and the clamping chains was calculated as 1.015. In the simulation verification test, the optimal parameter combination was used, and the optimal parameter combination was a garlic conveying speed of 0.8 m/s, an extension spring preload force of 16 N, and an extension spring stiffness of 215 N/m. After the above parameters were set, the simulation verification test was carried out.

Through simulation verification test, it was determined that the maximum floating displacement of the cutting component was 3.74 mm and the maximum angular velocity of swing arm reset was 57.93 deg/s under the condition of the optimal parameter combination. The orthogonal test results of groups 1-9 in **Table 2** and the optimal parameter combination test results were selected to form 10 groups of test results, as shown in **Table 7**. Then, a fuzzy comprehensive evaluation of the 10 groups of test results was performed. Membership models of the maximum floating displacement of the cutting component and the maximum angular velocity of swing arm reset used for the 10 groups of test results in **Table 7** are shown in Equations (11) and (12), respectively. The membership values *s*_1_ *_n_* and *s*_2_ *_n_* were obtained from Equations (11) and (12), respectively, and are listed in **Table 7**. The fuzzy relationship matrix ***S_n_*** was constructed from the membership values *s*_1_ *_n_* and *s*_2_ *_n_* is shown in Equation (13).

**Table 7:** Comprehensive scores of floating cutting performance based on 10 groups of test results.

Parameter combination		Maximum Floating Displacement of The Cutting Component *l* (mm)	Membership values of the maximum floating displacement of the cutting component based on 10 groups of test results *s*_1_ *_n_*	Weight of the maximum floating displacement of the cutting component	Maximum Angular Velocity of Swing Arm Reset *ω* (deg·s^-1^)	Membership values of the maximum angular velocity of swing arm reset based on 10 groups of test results *s*_2_ *_n_*	Weight of the maximum angular velocity of swing arm reset	Comprehensive scores based on 10 groups of test results *V*
Orthogonal test parameter combinations in **Table 2**	1	4.45	0.671	0.6	45.50	0.000	0.4	0.403
	2	5.16	0.343		46.49	0.076		0.236
	3	5.90	0.000		47.13	0.125		0.050
	4	4.78	0.519		52.01	0.498		0.510
	5	5.45	0.208		52.06	0.502		0.326
	6	4.03	0.866		52.94	0.569		0.747
	7	5.15	0.347		56.43	0.836		0.543
	8	3.81	0.968		57.29	0.901		0.941
	9	4.39	0.699		58.58	1.000		0.819
Optimal parameter combination	10	3.74	1.000		57.93	0.950		0.980

The 10 groups of test results, i.e., the test results of the optimal parameter combination and the test results of 9 groups of orthogonal tests in **Table 2**; Parameter combinations 1-9 corresponded to orthogonal test parameter combinations 1-9 in **Table 2**, respectively; Parameter combination 10 was the optimal parameter combination.


(11) $$s_{1n}=\frac{{l^{\prime }}_{\max}-{l^{\prime }}_{n}}{{l^{\prime }}_{\max}-{l^{\prime }}_{\min}}\left(n=1,2,\ldots .10\right)$$

(12) $$s_{2n}=\frac{{\omega^{\prime }}_{n}-{\omega^{\prime }}_{\min}}{{\omega^{\prime }}_{\max}-{\omega^{\prime }}_{\min}}\left(n=1,2,\ldots .10\right)$$

(13) $$S_{n}=\left(\begin{array}{c} s_{11}s_{12}s_{13}s_{14}s_{15}s_{16}s_{17}s_{18}s_{19}s_{110}\\ s_{21}s_{22}s_{23}s_{24}s_{25}s_{26}s_{27}s_{28}s_{29}s_{210} \end{array}\right)$$

Where, *s*_1_ *_n_* and *s*_2_ *_n_* are the membership values of the maximum floating displacement *l* of the cutting component and the maximum angular velocity *ω* of swing arm reset for the *n*th test in **Table 7**, respectively; *l′*_max_ and *l′*_min_ are the maximum and minimum values of index *l* in **Table 7**; *l′_n_* is the value of index *l* for the *n*th test in **Table 7**; *ω′*_max_ and *ω′*_min_ are the maximum and minimum values of index *ω* in **Table 7**; *ω′_n_* is the value of index *ω* for the *n*th test in **Table 7**; *n* is the test number; *s*_11_-*s*_110_ are the membership values of the maximum floating displacement of the cutting component for tests of groups 1-10 in **Table 7**, respectively; *s*_21_-*s*_210_ are the membership values of the maximum angular velocity of swing arm reset for tests of groups 1-10 in **Table 7**, respectively.

Same as the above virtual orthogonal test, the weight of the maximum floating displacement of the cutting component was set as 0.6 and the weight of the maximum angular velocity of swing arm reset was set as 0.4. Thus, the weight assignment set ***M*** was constructed as ***M*** = [0.6 0.4]. By fuzzy transformation, we get the comprehensive score set ***V***, where ***V*** = ***M*** · ***S*** *_n_*. Through the above calculations, the comprehensive scores of floating cutting performance for 10 groups of test were obtained, as listed in **Table 7**. As can be seen from **Table 7**, the comprehensive score of the optimal parameter combination was 0.980, which was higher than the comprehensive scores of the other 9 groups of orthogonal tests. The floating cutting performance of the optimized root-cutting mechanism was better than other parameter combinations. Therefore, the comprehensive optimization results are reliable.

### 3.3 Field verification test

#### 3.3.1 Test condition

A test bench of the garlic root-cutting mechanism was constructed to conduct a field verification test, with the purpose of verifying the accuracy of the numerical simulation model and reliability of the optimal parameter combination. The test bench is shown in **Figure 11**, in which each component is individually driven by speed-controlled motors. Parameters, such as the tilt angle and height of the test stand could be adjusted as required. Garlic plants were obtained from an experimental field in Jinxiang County, Shandong Province, China.

**Figure 11:** Test bench of garlic root-cutting mechanism.

#### 3.3.2 Design and scheme of field verification test

The two indexes assessed in the simulation tests, such as the maximum floating displacement of the cutting component and maximum angular velocity of swing arm reset, correspond to the root excision rate, which is the actual index of the root-cutting quality. The smaller the maximum floating displacement of the cutting component and the greater the angular velocity of swing arm reset, the easier it is to ensure that the protective fence was closely attached to the lower bulb surface for the floating root-cutting process. In this way, the cutting edge is close to the root disc of the garlic, the remaining length of the root after cutting is shorter, and the root excision rate is higher. Therefore, the field verification tests were conducted for nine parameter combinations of the virtual orthogonal test listed in **Table 2** and the optimal parameter combination in Section 3.2.3, using the root excision rate as the root-cutting quality index. The field verification tests were conducted sequentially for the nine parameter combinations listed in **Table 2**.

The garlic plants selected for the test were characterized by good uprightness, well-developed roots, and uniform bulb maturity. Before the tests, the garlic plants were tidied up and cleaned up to remove residual film, large pieces of soil, and debris on the roots. Each test was fed 90 garlic plants, and repeated three times for each parameter combination. The root excision rate was measured in the three tests, and the average value of the three tests was taken as the test result.

The root excision rate is the ratio of the total mass of the roots removed to the total mass of all roots. The root excision rate equation is expressed as:


(14) $$P=Q_{1}/\left(Q_{1}+Q_{2}\right)$$

where, *P* is the root excision rate (%); *Q*_1_ is the total mass of removed roots (g); *Q*_2_ is the total mass of remaining roots (g). Before weighing, the soil and debris on the root were also removed.

#### 3.3.3 Results and analysis of field verification test

The results of the verification test are summarized in **Table 8**. Using IBM SPSS Statistics 22 software, the data processing and statistical analysis of the test results were performed.

**Table 8:** Test schemes and results of field verification test.

Test number		Extension Spring Preload Force *A*	Extension Spring Stiffness *B*	Garlic Conveying Speed *C*	Root excision rate *P* (%)
1		1(14)	1(115)	1(0.8)	85.03
2		1(14)	2(165)	2(0.9)	83.77
3		1(14)	3(215)	3(1.0)	81.96
4		2(15)	1(115)	2(0.9)	87.61
5		2(15)	2(165)	3(1.0)	85.32
6		2(15)	3(215)	1(0.8)	90.56
7		3(16)	1(115)	3(1.0)	88.23
8		3(16)	2(165)	1(0.8)	92.37
9		3(16)	3(215)	2(0.9)	91.05
Root excision rate *P*	*K*_1_	250.76	260.87	267.96	
	*K*_2_	263.49	261.46	262.43	
	*K*_3_	271.65	263.57	255.51	
	Range	20.89	2.7	12.45	
	Significance Sequence of Factors *A>C>B* Optimal Parameter Combination *A*_3_ *C*_1_ *B*_3_				

K_31_~K_33_ were the sum of the root excision rate for a factor at level 1, level 2 and level 3, respectively.

The Shapiro-Wilk test was performed for the root excision rate in **Table 8**. The *P* value of the Shapiro-Wilk test was 0.788 (*P* > 0.05). The results indicate that the root excision rate obtained from 9 groups of field verification tests conformed to a normal distribution. Range analysis was performed on the test results, and the results are listed in **Table 8**. The significance of the factors affecting the root excision rate decreased in the following order: extension spring preload force, garlic conveying speed, and extension spring stiffness. The optimal parameter combination was *A*_3_ *C*_1_ *B*_3_. Based on the range analysis results, a radar diagram that was drawn to visually describe the effects of factors on the root excision rate is shown in **Figure 12**. As seen from **Figure 12**, the root excision rate was positively correlated with the extension spring preload force and stiffness and negatively correlated with the garlic conveying speed. ANOVA was performed on the test results. The ANOVA results are shown in **Table 9**. At the 95% confidence level, the effect of the extension spring preload force and garlic conveying speed on the root excision rate was highly significant (*P*< 0.01), and the effects of extension spring stiffness on the root excision rate were not significant (*P* > 0.05).

**Figure 12:** Effects of factors on the root excision rate. The nine radial axes in the figure were the root excision rate.

**Table 9:** ANOVA of field verification test.

Source	Sum of Squares	D*f*	Mean Squares	*F* Value	*P* Value
Extension Spring Preload Force *A*	73.892	2	36.946	328.963	0.0030
Extension Spring Stiffness *B*	1.343	2	0.672	5.981	0.1433
Garlic Conveying Speed *C*	25.941	2	12.971	115.488	0.0086
Error	0.225	2	0.112		

The comparison of the results of the virtual orthogonal and field verification tests showed that the optimal parameter combinations obtained from the two tests were the same. The influence law and significance of each factor on the root excision rate and comprehensive score for floating cutting performance were also the same. Thus, the accuracy of the numerical simulation model and the reliability of the simulation results were verified.

In order to verify the accuracy and reliability of the optimization results, the optimal parameter combination of *A*_3_ *C*_1_ *B*_3,_ which was optimized by the field verification tests, was used as the test condition to determine the root excision rate by the field test. To eliminate random errors, the test was repeated three times and the average value was taken as the test result. When the extension spring preload force was 16 N, garlic conveying speed was 0.8 m/s, and extension spring stiffness was 215 N/m, the root excision rate was 92.72% as measured in the field test.The test result (i.e., root cutting rate of 92.72%) was better than those of the other nine orthogonal test schemes listed in **Table 8**, which meets the requirements of Chinese garlic field harvesting quality. The bulbs after root-cutting are shown in **Figure 13**. Therefore, the optimal parameter combination *C*_1_ *A*_3_ *B*_3_ is reliable.

**Figure 13:** The bulbs after root-cutting.

In addition, the bulb damage caused by the cutting operation was studied by theoretical analysis in Section 2.3. To comprehensively assess the applicability and reliability of the optimal parameter combination for the root-cutting mechanism, the bulb damage rate during the cutting operation was tested. The test was repeated three times and the average value was taken as the test result. Under the optimal parameter combination, the average value of bulb damage rate was less than 6.0%, which meets the requirements of Chinese garlic field harvesting quality.

## 4 Discussion

In this study, the kinematic characteristics of the floating cutting process of the root-cutting mechanism, and technical methods for improving the root excision rate were investigated in detail. The optimal parameter combination for root-cutting mechanism was obtained through simulation analysis and verified by simulation and field tests. Based on kinematic analysis results of the floating process of the root-cutting mechanism and the pre-test results of the simulation, this study selected the extension spring preload force, extension spring stiffness, and garlic conveying speed as the test factors to carry out the simulation analysis, and devoted to investigate the influence law of each factor on the floating cutting performance and its formation causes. The effects of the different garlic varieties, different bulb sizes, and garlic plant collapse on the floating cutting performance of the root-cutting mechanism were not further investigated because of the short garlic harvesting period in China. Therefore, all test results only apply to Jinxiang garlic with good uprightness and uniform bulb maturity. Factors such as garlic variety, plant growth, plant collapse, and the assembly with the combine harvester need to be further studied. In the next step, the root-cutting mechanism will be configured in the garlic combine harvester to perform field tests. The adaptability of the root-cutting mechanism to different garlic varieties, plant collapse and bulb maturity will be examined, and the root-cutting mechanism will be further optimized.

The tests showed that because there were only two protective fences between the bulb and rotary cutter group, the garlic roots easily passed through the protective fences and were fully cut by the rotary cutter group, resulting in a high root excision rate. At the same time, it was observed in the tests that the risk of cutting the bulb during the root-cutting process was effectively reduced by using protective fences that formed a physical barrier between the bulb and the rotary cutter group, which separates the bulb from the rotary cutter group. However, we found that the reliability of the rotary cutter group and protective fences still need to be further improved. After a long period of operation, the rotary cutter group was worn out, while the protective fences were deformed. In future product development, it is recommended that the rotary cutter group and the protective fences be made of high-quality high-speed steel and high quality spring steel respectively with strict heat treatment process to further improve the reliability of the root-cutting mechanism.

## 5 Conclusions

In response to the problems of technological backwardness and poor operational quality of mechanized root-cutting in garlic field harvesting in China, we combined the physical characteristics and agronomic requirements of garlic plants to develop a new floating root-cutting technology for garlic combine harvesters. The coordinate equations of the initial contact point of the bulb and a mathematical model of the floating displacement of the cutting component were established. Using computer simulation techniques, the influence law of the garlic conveying speed, extension spring preload force and stiffness on the floating cutting performance and its formation causes were analyzed, and the optimal parameter combination of the root-cutting mechanism was determined. The test results showed that the floating cutting performance was positively correlated with the extension spring preload force and stiffness and negatively correlated with the garlic conveying speed. Among them, the effects of extension spring preload force and garlic conveying speed on the floating cutting performance were highly significant. The simulation and field validation tests showed that the garlic floating root-cutting technology enabled the top alignment of bulb, adaptive profiling floating of cutter, and embedded cutting of roots and its technology scheme was feasible and effective and achieved the best operating performance. The floating cutting performance of the root-cutting mechanism met the requirements of Chinese garlic field harvesting quality.

## Data availability statement

The original contributions presented in the study are included in the article/supplementary material. Further inquiries can be directed to the corresponding authors.

## Author contributions

Conceptualization, MY and ZH. Methodology, FG. Formal analysis, BP. Data curation, KY. Writing—original draft preparation, ZY and KY. Writing—review and editing, ZY and YZ. All authors contributed to the article and approved the submitted version.
